The article "Clinical Outcomes of Cannulated Screws versus Ring Pin versus K-Wire with Tension Band Fixation Techniques in the Treatment of Transverse Patellar Fractures: A Case-Control Study with Minimum 2-Year Follow-Up" was published in 2022. Journal: Biomed Res Int.

# Clinical Outcomes of Cannulated Screws versus Ring Pin versus K-Wire with Tension Band Fixation Techniques in the Treatment of Transverse Patellar Fractures: A Case-Control Study with Minimum 2-Year Follow-Up

**DOI:** 10.1155/2022/5610627

**Published:** 2022-06-15

**Authors:** Junchuan Liu, Yiming Ge, Guolei Zhang, Xuehong Zheng, Liang Gao, Enzeng Xing, Jiangfeng Lu, Jun Di, Junfei Guo

**Affiliations:** ^1^Department of Orthopaedic Surgery, The Third Hospital of Hebei Medical University, Shijiazhuang, Hebei, China; ^2^Department of Psychiatry, Hebei Medical University, Shijiazhuang, China; ^3^Department of Orthopaedic Surgery, Hebei General Hospital, Shijiazhuang, Hebei, China; ^4^Department of Orthopaedic Surgery, The People's Hospital of Xinhe County, Xingtai, Hebei, China

## Abstract

**Purpose:**

K-wire with tension band (KTB) technique has long been the primary surgical method for transverse patella fractures; however, it also has shortcomings. This study is aimed at evaluating the three different techniques to see whether the cannulated screw tension band (CSTB) or ring pin tension band (RPTB) techniques could decrease complications and achieve better knee function compared with KTB.

**Methods:**

We conducted a retrospective comparison of the KTB, CSTB, and RPTB fixation techniques. We selected and reviewed 90 patients (30 patients in each fixation group) with follow-up at least 2 years. Duration of operation, intraoperative blood loss, mean healing time, visual analog scale score, range of motion, Böstman score, Iowa knee score, modified Lysholm rating scale, and postoperative complications were compared. Multivariate analyses were performed to identify the independent risk factors for fracture healing time, postoperative complications, and knee function recovery.

**Results:**

After adjusting for confounding factors, multivariate regression analysis revealed that CSTB was 0.26 times (95% CI: 0.08-0.86, *p* = 0.027) less likely to prolong fracture healing time, 0.20 times (95% CI: 0.06-0.64, *p* = 0.007) lesser risk of postoperative complications, and more than four times (95% CI: 1.41-13.56, *p* = 0.011) as likely to improve the knee function score compared with KTB. Besides, RPTB were also superior to KTB in reducing the incidence of postoperative complications (OR: 0.21, 95% CI: 0.07-0.64, *p* = 0.006) and improved knee function score (OR: 3.96, 95% CI: 1.30-12.08, *p* = 0.016); however, the CSTB group being more superior. In addition, AO/OTA C2 fractures (OR, odds ratio: 10.68, 95% CI: 1.30-87.70, *p* = 0.027) and high-energy fracture (OR: 8.78, 95% CI: 1.57-49.17, *p* = 0.013) were also associated with prolonged fracture healing time but not with postoperative complications and knee function. No significant differences in related indicators such as gender, age, BMI, AO/OTA classification, fracture side, injury mechanism, duration of operation, and intraoperative blood loss were detected among the three groups.

The article "Clinical Outcomes of Cannulated Screws versus Ring Pin versus K-Wire with Tension Band Fixation Techniques in the Treatment of Transverse Patellar Fractures: A Case-Control Study with Minimum 2-Year Follow-Up" was published in 2022. Journal: Biomed Res Int.

**Conclusion:**

This study demonstrated that the CSTB technique is superior to KTB and RPTB techniques in reducing the incidence of postoperative complications, and it also has advantages in accelerating fracture healing, achieving better VAS, ROM, and functional recovery. Further long-term large-sized prospective randomized trials are needed to evaluate the efficacy of the KTB in treating transverse patellar fractures.

## 1. Introduction

With the rapid development of social and economic undertakings, the number of patellar fractures caused by high-energy trauma, such as falling from high places, industrial production, and traffic accidents, is increasing, which accounts for approximately 1% of all skeletal system fractures [1, 2]. The patella plays an essential role in knee function, with a primary function to increase quadriceps muscle strength and maintain the extension of the knee joint. In addition, the intact patella is an important barrier that protects the knee from external damage. As a common fracture type, clinically, patella fracture may lead to decreases of quadriceps muscle strength [3] and range of motion (ROM) of the knee joint [4, 5] and traumatic arthritis [6, 7], which has a serious impact on the health and quality of life of the patients.

At present, the primary and conventional surgical method for the treatment of patellar transverse fracture is surgical fixation with K-wire tension band (KTB), which has been firstly defined by Müller et al. in 1979 [8]. The technical advantage of this standard technique is that this method can convert tension at the fracture site, which is produced by tension band fixation into compression forces at the articular surface, helping in accelerating the healing of the fracture [9, 10]. This technique has been widely accepted by orthopaedic trauma surgeons because of its reliable fixation, allowance of early joint motion, and mostly achieving the goals that provide a congruent articular surface and maintain rigid fixation [11, 12]. However, a number of studies showed a significant incidence of postoperative complications, including pain, infection, wire breakage, migration, and reduction loss, making the best surgical approach remaining controversial when considering fixation using cannulated screws tension band (CSTB) or ring pins with supplementary tension band (RPTB) [13–20]. Additionally, overall long-time functional recovery after surgery is still less than satisfactory [7].

The article "Clinical Outcomes of Cannulated Screws versus Ring Pin versus K-Wire with Tension Band Fixation Techniques in the Treatment of Transverse Patellar Fractures: A Case-Control Study with Minimum 2-Year Follow-Up" was published in 2022. Journal: Biomed Res Int.

Controversy exists within the previous literature regarding the optimal fixation technique for transverse patellar fractures. Zhu et al. and Tian et al. concluded in their respective studies that CSTB is superior to KTB [1, 15]. However, Hoshino et al. [21] found there was a trend towards significantly more fixation failures with CSTB compared to KTB, although CSTB decreased the prevalence of symptomatic hardware. Tian et al. [15] found that the Iowa knee score was significantly improved in the CSTB group, while Wang et al. found there was no significant difference in the same score between the two groups [22]. In terms of the postoperative functional recovery time and pain relief effects, literature results are also controversial [13, 14, 16]. Thus, the objective of the present study was to evaluate the three different tension-band techniques to see whether CSTB or RPTB techniques could (1) shorten fracture healing time, (2) decrease complications, and (3) achieve better knee function compared with KTB.

## 2. Materials and Methods

### 2.1. Patients and Groups

After approval from the Institutional Review Committee of our hospital and obtained the informed written consent from all patients in accordance with the Declaration of Helsinki, we performed a retrospective cohort study from August 2017 to May 2019. We included 30 patients who were treated with open reduction and fixation with the KTB approach in the KTB group. To improve the reliability of the current research, we used a 1 : 1 : 1 ratio regarding age, sex, body mass index (BMI), fracture side, injury mechanism, and AO/OTA classification [23] to select 30 patients, respectively, who underwent CSTB and RPTB approach for comparisons (Figure 1). Operations were considered when the articular displacement was greater than 2 mm or fragment separation was greater than 3 mm on radiography. Patient selections were influenced by cost as the CSTB and RPTB techniques were offered only to patients who agreed to pay for this higher-cost procedure.

The inclusion criteria were (1) aged 18 years and above; (2) patients diagnosed with unilateral transverse patella fracture: AO/OTA 34-C1 fractures and AO/OTA 34-C2 fractures; (3) patients with enclosed injuries; (4) patients who underwent surgical stabilization with KTB, CSTB, or RPTB techniques; and (5) patients had relatively complete research data. Exclusion criteria were aged younger than 18 years, the presence of open fractures, the presence of concomitant fractures, patients who had stiff knee or other function limitation of the knee, previous open knee surgery, neurological problems, and declining to participate.

The article "Clinical Outcomes of Cannulated Screws versus Ring Pin versus K-Wire with Tension Band Fixation Techniques in the Treatment of Transverse Patellar Fractures: A Case-Control Study with Minimum 2-Year Follow-Up" was published in 2022. Journal: Biomed Res Int.

### 2.2. Surgical Procedures

All patients received the same anesthesia, and all surgeries were performed by the same senior orthopedic surgeon. All patients received a single dose of a first-generation cephalosporin antibiotic for prophylaxis, or if allergic, the type of specific antibiotic used depended on the surgeon's preference. The selection of KTB (Figures 2(a)–2(f)), CSTB (Figures 3(a)–3(f)), or RPTB (Figures 4(a)–4(f)) were based on the surgeon's preference and patient's willingness and economic income. In each group, all surgeries were performed via an anterior longitudinal incision. After sectioning the skin and subcutaneous tissue followed by fully exposing the patella, we examined the fracture and condition of the bilateral aponeuroses and joint capsule, removed the fracture chips and intra-articular hematoma, then rinsed the articular cavity. Supplementary fixation, including interfragmentary cannulated screw, cable pins, or K-wires, was used if necessary. Stability of fracture fixation was confirmed with the knee in flexion of at least 90 degrees. Position of internal fixation and ROM of the joint were checked as well before closing the incision. After surgery, the wound was closed in a standard layered fashion, and none of the cases had an articular step greater than 1 mm or an interfragmentary gap greater than 2 mm on postoperative radiography.

### 2.3. Postoperative Treatment

All participants received the same postoperative pain control and rehabilitation programs. All patients performed quadriceps contraction exercises immediately after the surgery; passive joint flexion and extension exercises were best started on the second day, and active joint flexion and extension exercises were allowed and encouraged 7 days after the operation. One month later, patients were permitted to perform partial weight-bearing walking, while performing full weight-bearing walking two months after the operation.

### 2.4. Outcome Measures

Assessments were performed by a senior orthopedic surgeon who did not involve in patient treatments. Parameters including duration of operation, intraoperative blood loss, visual analog scale (VAS), ROM, Böstman score [24, 25], Iowa knee score [26], and modified Lysholm rating scale [27, 28], fracture healing time, and postoperative complications (fixation failure, implant breakage or loosening, painful hardware, infection, and skin breakdown) for all patients were recorded or assessed. All patients' conventional radiographs were obtained at 1, 3, 6, 12, 18, and 24 months after the operation to assess the fracture healing status. The ROM, Böstman score, Iowa knee score, and modified Lysholm rating scale were evaluated at 6 months after the operation to ensure a uniform, standardized evaluation and assessment. Both the radiographic and clinical union were used to define fracture healing, as when a patient had no local pain or tenderness, the ability to walk well without help, and as the fracture lines became blurred with a continuous callus passing through it.

The article "Clinical Outcomes of Cannulated Screws versus Ring Pin versus K-Wire with Tension Band Fixation Techniques in the Treatment of Transverse Patellar Fractures: A Case-Control Study with Minimum 2-Year Follow-Up" was published in 2022. Journal: Biomed Res Int.

In terms of complications, fixation failure was defined as a loss of reduction before bone healing and required revision. Infection was defined as that occurred before wound healing, while skin breakdown was defined as a secondary skin lesion after the initial wound healing.

### 2.5. Statistical Analysis

We performed a power analysis for the statistics. A two-sided 5% significance level and 80% power were considered as reliable and significant. The sample size and power analysis have been computed using NCSS-PASS V11.0.7 software (https://www.ncss.com/software/pass/). The continuous variables were evaluated for normality by using the Shapiro-Wilk test. Data satisfying normality are presented as the mean ± standard deviation. The tests for significant differences between normally distributed data samples were performed using Student's *t*-test. Categorical data are presented as absolute numbers (percentages), and the Chi-square or Fisher's exact tests were used to compare patient number distributions between the groups. Logistic regression was used to determine whether age, gender, BMI, AO/OTA classification, fracture side, injury mechanism, and type of fixation technique influenced the differences among the three groups in terms of fracture healing time, postoperative complications, and knee function recovery. All data analyses were performed using the IBM SPSS Statistics for Windows, version 26.0 (IBM, Armonk, NY, USA). The level of significance was set at *p* < 0.05.

## 3. Results

Patient demographics, injury-related data, and outcomes of the three groups are summarized in Tables 1 and 2. There were 30 patients in each group: 21 men and 9 women with a mean age of 46.7 years (range, 20–68 years) in the KTB group, 20 men and 10 women with a mean age of 43.2 years (range, 20–68 years) in the CSTB group, and 22 men and 8 women with a mean age of 43.0 years (range, 20–66 years) in RPTB group. All patients were followed up for at least 2 years, and none of the patients was lost to follow-up. No significant differences were found for demographics and injury-related data among the three groups (all *p* > 0.05, Table 1).

Table 2 showed that there was no difference (*p* > 0.05) in the duration of operation and intraoperative blood loss among the three groups. Although the mean healing time did not differ among the three groups, post hoc analysis revealed that the mean fracture healing time was shorter in the CSTB group than in the KTB group (2.1 months versus 2.3 months, *p* = 0.029). We found significant differences regarding the VAS and ROM, which were better in the CSTB group than those in the KTB and RPTB groups (all *p* < 0.001). In addition, all involved knee function scores were better in the CSTB group than the other two groups. In terms of postoperative complications, the incidence of implant breakage or loosening and painful hardware were significantly lower in the CSTB group, while fixation failure, infection, and skin breakdown did not reach a significant difference (Table 2).

The article "Clinical Outcomes of Cannulated Screws versus Ring Pin versus K-Wire with Tension Band Fixation Techniques in the Treatment of Transverse Patellar Fractures: A Case-Control Study with Minimum 2-Year Follow-Up" was published in 2022. Journal: Biomed Res Int.

The results of logistic regression analysis demonstrated that AO/OTA C2 fractures (OR, odds ratio: 10.68, 95% CI: 1.30-87.70, *p* = 0.027) and high-energy fracture (OR: 8.78, 95% CI: 1.57-49.17, *p* = 0.013) were associated with prolonged fracture healing time but not with postoperative complications and knee function. Our results showed that patients who underwent CSTB fixation were 0.26 times less likely to prolong fracture healing time compared with KTB (OR: 0.26, 95% CI: 0.08-0.86, *p* = 0.027). Besides this, the treatments of both CSTB and RPTB were superior to KTB in reducing the incidence of postoperative complications (OR: 0.20, 95% CI: 0.06-0.64, *p* = 0.007, and OR: 0.21, 95% CI: 0.07-0.64, *p* = 0.006, respectively) and improved knee function score (OR: 4.37, 95% CI: 1.41-13.56, *p* = 0.011, and OR: 3.96, 95% CI: 1.30-12.08, *p* = 0.016, respectively), with the CSTB group being more superior. Meanwhile, no significant difference in related indicators such as gender, age, BMI, AO/OTA classification, fracture side, and injury mechanism was detected (Table 3).

## 4. Discussion

Patellar fractures account for around 1% of all human body fractures, mainly in adults of 20–50 years old. Open reduction and various internal fixations can be applied clinically to reconstruct the anatomical structure and recover the function, such as KTB, CSTB, and RPTB, where the most widely accepted surgical method for the treatment of transverse patellar fracture is KTB [11, 12, 19, 29].

Despite the multitude of investigations being present in the literature, controversy in this field regarding the favorable choice of the device remains. It is generally known that applying an optimal technique not only requires shortening the fracture healing time and achieving better function but also reducing the postoperative complications. Compared with conventional techniques, the present study showed CSTB may not only serve as a favorable surgical technique with rare hardware irritation, implant breakage, and loosening but also provide continuous compression to accelerate fracture healing, thereby permitting an early postoperative functional recovery with a low incidence of postoperative complications. Taken together, the findings of this study showed that the CSTB technique is superior to both RPTB and traditional KTB techniques in the treatment of transverse patella fractures, which are in accordance with conclusions both from a high-quality meta-analysis [29] and laboratory biomechanical studies [30–32].

The article "Clinical Outcomes of Cannulated Screws versus Ring Pin versus K-Wire with Tension Band Fixation Techniques in the Treatment of Transverse Patellar Fractures: A Case-Control Study with Minimum 2-Year Follow-Up" was published in 2022. Journal: Biomed Res Int.

In terms of the mechanism of primary pressure achieved, there are differences among the three techniques. Compared with CSTB fixation, KTB and RPTB do not generate reduction and compression effects on the fragments directly. Instead, the compression effects on the patella are mainly exerted by tightening the wires or cables [33]. The failure mechanism with tension band wiring was reported due to slippage of the cerclage wire and then sinking of the K-wire into the patella [12], while that with CSTB may partly due to the difficulty in appropriate insertion of cannulated screws [34]. Notably, the incidence of fixation failure in CSTB is more than twice of that in KTB group (5/30 versus 2/30) according to our results. The difference did not, however, reach a statistical significant level, which may be due to the small number of samples; yet, a statistical trend was shown. This conclusion is similar to Hoshino et al. [21], who also observed a trend toward higher fixation failures with the use of CSTB compared to KTB.

As another two predominant obstacles troubling clinical doctors and limiting the outcome of patella fracture patients, implant breakage/loosening and painful hardware often require secondary surgery, which not only increases economic costs but also brings additional trauma to the patients. In the current study, the incidence of implant breakage/loosening and painful hardware in the CSTB group was the lowest among the three groups. Our multiple regression analysis indicated that the CSTB technique has positive effects on healing time, postoperative complications, and knee function recovery. With respect to the healing time, AO/OTA type and injury mechanism were another two independent risk factors, which is aligned with the previous research [15]. Given that other postoperative complications, like infection and skin breakdown, were negligible with a quite homogeneous distribution among the groups, taken together, we conclude that the CSTB technique is superior to KTB and RPTB techniques.

To the best of our knowledge, the superiority of the CSTB technique may be attributed to the following two reasons: (1) compared with the conventional KTB technique, CSTB is minimally invasive with a smaller incision and less soft tissue dissection, allowing early mobilization and faster recovery; (2) biomechanical studies have revealed that the screw fixation system may provide not only more stable and rigid fixation but also higher resistance against the distraction forces than the tension band wiring [35, 36]; (3) the CSTB technique could contact the bone surface more tightly, then provides more compression [16].

The article "Clinical Outcomes of Cannulated Screws versus Ring Pin versus K-Wire with Tension Band Fixation Techniques in the Treatment of Transverse Patellar Fractures: A Case-Control Study with Minimum 2-Year Follow-Up" was published in 2022. Journal: Biomed Res Int.

There are several limitations associated with our study. First, the data was collected in a single center with a relative small number of samples. Second, the decision to treat patients with what approach was subject to selection bias as this was not a randomized study. Third, although we controlled many possible confounding variables by multivariate regression, endogeneity bias from other omitted variables such as bone density, which may affect the results of the current study. Finally, the degree tightened in the titanium cable or the steel wire was not standardized to ensure that the tension was equal in any of the patients; however, each cohort of patients received the same surgery by the same orthopedic surgeon (JCL), which eliminated the effects of possible confounding variables.

## 5. Conclusion

This study demonstrated that the CSTB technique is superior to KTB and RPTB techniques in reducing the incidence of postoperative complications, and it also has advantages in accelerating fracture healing, achieving better VAS, ROM, and functional recovery. Further long-term large-sized prospective randomized trials are needed to evaluate the efficacy of the KTB in treating transverse patellar fractures.

## Figures and Tables

**Figure 1:** Flow chart of the study participants.

**Figure 2:** (a–f) A 44-year-old man with a transverse patellar fracture had K-wire tension band fixation. (a) An anteroposterior X-ray shows the transverse patellar fracture after injury. (b) A lateral X-ray after injury. (c) A postoperative anteroposterior X-ray of 1 month. (d) A postoperative lateral X-ray of 1 month. (e) A postoperative anteroposterior X-ray of 6 months. (f) A postoperative lateral X-ray of 6 months.

**Figure 3:** (a–f) A 37-year-old man with a transverse patellar fracture had cannulated screws tension band fixation. (a) An anteroposterior X-ray shows the transverse patellar fracture after injury. (b) A lateral X-ray after injury. (c) A postoperative anteroposterior X-ray of 1 month. (d) A postoperative lateral X-ray of 1 month. (e) A postoperative anteroposterior X-ray of 6 months. (f) A postoperative lateral X-ray of 6 months.

**Figure 4:** (a–f) A 54-year-old woman with a transverse patellar fracture had ring pin tension band fixation. (a) An anteroposterior X-ray shows the transverse patellar fracture after injury. (b) A lateral X-ray after injury. (c) A postoperative anteroposterior X-ray of 1 month. (d) A postoperative lateral X-ray of 1 month. (e) A postoperative anteroposterior X-ray of 6 months. (f) A postoperative lateral X-ray.

The article "Clinical Outcomes of Cannulated Screws versus Ring Pin versus K-Wire with Tension Band Fixation Techniques in the Treatment of Transverse Patellar Fractures: A Case-Control Study with Minimum 2-Year Follow-Up" was published in 2022. Journal: Biomed Res Int.

**Table 1:** Demographics and injury-related data of 90 study participants, stratified by fixation type.

Characteristics	KTB (*n* = 30)	CSTB (*n* = 30)	RPTB (*n* = 30)	*p* value
Demographic				
Age, years	46.7 ± 12.5	43.2 ± 13.4	43.0 ± 13.5	0.476
Gender				0.853
Male	21 (70.0%)	20 (66.7%)	22 (73.3%)	
Female	9 (30.0%)	10 (33.3%)	8 (26.7%)	
BMI group, no. (%)				0.600
Normal (BMI < 24 kg/m^2^)	10 (33.3%)	12 (40.0%)	13 (43.3%)	
Overweight (24 ≤ BMI < 28 kg/m^2^)	17 (56.7%)	16 (53.3%)	12 (40.0%)	
Obesity (BMI ≥ 28 kg/m^2^)	3 (10.0%)	2 (6.7%)	5 (16.7%)	
Injury-related data				
AO/OTA classification				0.506
34-C1	24 (80.0%)	20 (66.7%)	22 (73.3%)	
34-C2	6 (20.0%)	10 (33.3%)	8 (26.7%)	
Fracture side				0.561
Left	18 (60.0%)	15 (50.0%)	14 (46.7%)	
Right	12 (40.0%)	15 (50.0%)	16 (53.3%)	
Injury mechanism, no. (%)				0.539
Low-energy fracture	27 (90.0%)	25 (83.3%)	24 (80.0%)	
High-energy fracture	3 (10.0%)	5 (16.7%)	6 (20.0%)	

KTB: K-wire with tension band; CSTB: cannulated screws with tension band; CPTB: cable pin with tension band; BMI: body mass index. Values are presented as the number (%). Age is presented as the mean ± standard deviation.

**Table 2:** Clinical and functional outcomes, stratified by fixation type.

Characteristics	KTB (*n* = 30)	CSTB (*n* = 30)	RPTB (*n* = 30)	*p* value
Duration of operation	58.5 ± 6.3	56.5 ± 11.1	58.2 ± 7.0	0.615
Intraoperative blood loss	83.0 ± 12.6	84.0 ± 14.5	79.7 ± 12.0	0.411
Mean healing time (months)	2.3 ± 0.3^#^	2.1 ± 0.3	2.2 ± 0.2	0.081
VAS	3.8 ± 0.8^¶^	2.8 ± 0.9	3.6 ± 0.9^¶^	<0.001^∗^
ROM	105.1 ± 3.8^&^	112.2 ± 6.3	107.4 ± 4.5^&^	<0.001^∗^
Böstman score				0.037^∗^
28-30	21 (30.0%)	29 (96.7%)	26 (86.7%)	
20-27	5 (16.7%)	1 (3.3%)	3 (10.0%)	
<20	4 (13.3%)	0 (0.0%)	1 (3.3%)	
Iowa knee score				0.023^∗^
90-100	17 (56.7%)	28 (93.3%)	23 (76.7%)	
80-89	6 (20.0%)	2 (6.7%)	4 (13.3%)	
70-79	4 (13.3%)	0 (0.0%)	2 (6.7%)	
<70	3 (10.0%)	0 (0.0%)	1 (3.3%)	
Modified Lysholm rating scale	83.7 ± 11.9	92.2 ± 7.7^^^	89.7 ± 9.6^^^	0.004^∗^
Postoperative complications				
Fixation failure	2 (6.7%)	5 (16.7%)	1 (3.3%)	0.174
Implant breakage or loosening	13 (43.3%)	3 (10.0%)	5 (16.7%)	0.005^∗^
Painful hardware	11 (36.7%)	1 (3.3%)	3 (10.0%)	0.001^∗^
Infection	3 (10.0%)	0 (0.0%)	1 (3.3%)	0.108
Skin breakdown	1 (3.3%)	0 (0.0%)	0 (0.0%)	0.330

KTB: K-wire with tension band; CSTB: cannulated screws with tension band; CPTB: cable pin with tension band; VAS: visual analog scale; ROM: range of motion. Values are presented as the number (%). Duration of operation, intraoperative blood loss, mean healing time, VAS, ROM, and modified Lysholm rating scale are presented as the mean ± standard deviation. ^∗^*p* < 0.05, statistical significance. ^#^Significant differences in statistics compared with CSTB group (*p* = 0.0029). ^¶^Significant differences in statistics compared with CSTB group (all *p* < 0.001). ^&^Significant differences in statistics compared with CSTB group (all *p* < 0.001). ^^^Significant differences in statistics compared with KTB group (all *p* < 0.05).

The article "Clinical Outcomes of Cannulated Screws versus Ring Pin versus K-Wire with Tension Band Fixation Techniques in the Treatment of Transverse Patellar Fractures: A Case-Control Study with Minimum 2-Year Follow-Up" was published in 2022. Journal: Biomed Res Int.

**Table 3:** Results of multivariate logistic regression analysis.

Variable (reference)	Fracture healing time			Postoperative complications			Knee function		
	OR	95% CI	*p* value	OR	95% CI	*p* value	OR	95% CI	*p* value
Gender (male)	2.01	0.64-6.35	0.234	0.56	0.20-1.63	0.289	1.12	0.38-3.24	0.840
Age (≤40)	1.18	0.40-3.52	0.766	0.92	0.33-2.57	0.870	0.62	0.22-1.81	0.384
BMI (normal)									
Overweight	1.23	0.42-3.56	0.707	1.58	0.33-7.58	0.568	0.64	0.13-3.03	0.571
Obesity	1.04	0.21-5.21	0.965	0.94	0.34-2.60	0.899	0.77	0.32-3.21	0.568
AO/OTA (34-C1)	10.68	1.30-87.70	0.027^∗^	2.12	0.37-12.03	0.397	0.48	0.08-3.04	0.434
Fracture side (left)	0.96	0.17-5.51	0.966	1.13	0.34-3.78	0.841	2.50	0.68-9.18	0.166
Injury mechanism (low-energy fracture)	8.78	1.57-49.17	0.013^∗^	0.27	0.04-1.70	0.162	1.64	0.25-10.84	0.607
Operation method (KTB)									
CSTB	0.26	0.08-0.86	0.027^∗^	0.20	0.06-0.64	0.007^∗^	4.37	1.41-13.56	0.011^∗^
RPTB	0.67	0.20-2.27	0.524	0.21	0.07-0.64	0.006^∗^	3.96	1.30-12.08	0.016^∗^

KTB: K-wire with tension band; CSTB: cannulated screws with tension band; CPTB: cable pin with tension band; BMI: body mass index. ^∗^*p* < 0.05, statistical significance.

## Data Availability

The data presented in this study are available on request from the corresponding author.

## Abbreviations

ROM: Range of motion
KTB: K-wire tension band
CSTB: Cannulated screws tension band
RPTB: Ring pin tension band
BMI: Body mass index
VAS: Visual analog scale.
